The article "The Role of Twitter Medium in Business with Regression Analysis and Statistical Modelling" was published in 2021. Journal: Comput Intell Neurosci.

# The Role of Twitter Medium in Business with Regression Analysis and Statistical Modelling

**DOI:** 10.1155/2021/1346994

**Published:** 2021-10-19

**Authors:** Jia Cong, Zubair Ahmad, Basim S. O. Alsaedi, Osama Abdulaziz Alamri, Ibrahim Alkhairy, Hassan Alsuhabi

**Affiliations:** ^1^Marketing Department, Management School, Lancaster University, Lancaster, UK; ^2^Department of Statistics, Yazd University, P.O. Box 89175-741, Yazd, Iran; ^3^Department of Statistics, Faculty of Science, University of Tabuk, Tabuk, Saudi Arabia; ^4^Department of Mathematics, Al-Qunfudah University College, Umm Al-Qura University, Mecca, Saudi Arabia

## Abstract

Marketing refers to the strategies a company undertakes to promote its brands to its potential audience. Advertising provides useful venues for marketing to promote a company's survives/goods to the audience. It has a positive impact on the sale of services or products. In this study, we consider a well-known online medium called Twitter (the fourth most popular social media platform used by marketers) to check its impact on sales. For this purpose, the simple linear regression modeling approach is implemented to test the significance and usefulness of Twitter advertising on sale. Statistical tests such as *t*-test and correlation test are adopted to test the hypothesis of the “impact of Twitter advertising on sales.” Based on the findings of this study, it is observed that Twitter advertising has a positive impact on sales. Furthermore, a new statistical model called the exponential T-X exponentiated exponential is introduced. The proposed model is very interesting and possesses heavy-tailed characteristics which are useful in finance and other related sectors. Finally, the applicability of the new model is illustrated by considering the sales data.

## 1. Introduction

Advertisement is a way of marketing to communicate with the potential consumers of certain goods, products, or services. Advertisements are the information usually paid by a company to influence consumer's decision to buy their products. Numerous mediums are available for advertisements and marketing. The available mediums can be divided into two main groups, such as printed mediums and online mediums. Online media is the most effective medium to reach more consumers [1, 2].

Online advertising is a way of marketing to convey messages to potential users via using the Internet. It is also called online marketing and helps in finding the potential and right audience. Online advertisements appear in a search engine, on social media, in a browser, or even in e-mail. Online advertising can be classified into different groups such as display ads, e-mail ads, native ads, video ads, and social media ads [3, 4].

The article "The Role of Twitter Medium in Business with Regression Analysis and Statistical Modelling" was published in 2021. Journal: Comput Intell Neurosci.

Twitter is one of the most prominent online/social media platforms that can be used quite effectively for advertising a particular brand. It is a fruitful tool for marketing the business and engaging the audience. It permits its users to create accounts and interact with others through short messages called “tweets.” Twitter is one of the marketer's favorite social media platforms. For instance, 53% of marketers worldwide used it as a channel for their marketing activities in 2020. Social media generally provides brands with personally consumer-related opportunities. Twitter has a huge impact on consumer behavior. According to a report by the Digital Marketing Institute, it turns out that about 40% of Twitter users bought something after seeing it on Twitter. This reflects the steadily increasing impact of social media on consumers' buying habits [5–8].

Not only is it enough to get the company brand involved on Twitter but also brands need to consider the facilities of social media influencers. The influence of social media like Twitter is also competing with friends in building consumer trust. When trying to find a product recommendation, 56% of consumers asked their friends for instructions, and 49% of respondents said that they bought something after consulting their friends; see [9]. On Twitter, recommendations from influencers resulted in a 20% increase in the sale of products [10]. It is ranked fourth in the marketing arena; see Figure 1.

In this paper, we analyze a real-life data set related to Twitter advertising to see its impact on sales. We will use a well-known statistical methodology called the regression technique to see how much the sales can be increased by spending money on Twitter advertising. To carry out the regression analysis, we will test the hypothesis of “the impact of Twitter advertising on sales.” In this regard, the null hypothesis (NH) expressed by *H*_0_ and alternative hypothesis (AH) denoted by *H*_*A*_ will be formulated as follows: *H*_0_ = Twitter advertising has no significant impact on sales versus *H*_*A*_ = Twitter advertising has a significant impact on sales.

Furthermore, to provide an adequate fit to the sales data, a new heavy-tailed (HT) statistical model is introduced. The new model is introduced by combining the exponential distribution with the exponential TX strategy. The new model is entitled the exponential T-X exponentiated exponential (ETXE-exponential) model. The comparison of the ETXE-exponential distribution is done with the other models. The numerical results show that the ETXE-exponential is a suitable model for dealing with data in business, finance, and management sciences.

The article "The Role of Twitter Medium in Business with Regression Analysis and Statistical Modelling" was published in 2021. Journal: Comput Intell Neurosci.

## 2. Regression Analysis

The regression method helps to carry out the regression analysis to forecast the demand for a particular product. It determines the nature of the relationship between the product's demand and its corresponding determinants. The regression analysis can be carried out via three main approaches, depending upon the nature of the study.  Figure 2 illustrates the main divisions of the regression analysis.

### 2.1. Simple Linear Regression Approach

In this paper, we adopt the simple linear regression (SLReg) approach as we have one independent variable (Twitter advertisement). This approach helps to predict the response variable, usually represented by *Y* based on the independent variable(s) usually represented by *X*. The simple linear regression can be expressed mathematically as follows:

(1) $$\begin{array}{c} Y=\theta_{0}+\theta_{1}X+\varepsilon , \end{array}$$

where *θ*_0_ is representing the intercept of the model and *θ*_1_ is called the slope of the model. A value 0 of *θ*_1_ indicates no effect of *X* on *Y*, and in such situation, the model is given by *Y*=*θ*_0_. The quantity *ε* is the residual error term having a mean value of 0.

In case of explaining the relationship between sales *Y* and Twitter advertising *X*, the simple linear regression becomes

(2) $$\begin{array}{c} \text{Sales}=\theta_{0}+\theta_{1}\text{Twitter}+\varepsilon . \end{array}$$

After carrying out the analysis using the regression technique, we found that *θ*_0_=5.621 representing the predicted sales in thousands of USD (United States dollars), when there is no investment on the Twitter medium. Therefore, under the circumstances of no investment on Twitter medium, the expected sale would be 5.621*∗*1000=5621 dollars.

The slope (also called the regression coefficient) of the regression model *θ*_1_, provided in equation (2), is 0.193 representing 193(0.193*∗*100) units increment in the sales. Henceforth, using the Twitter medium as a marketing tool, the predicted/estimated sale is 5.621+0.193*∗*1000=198.621, representing a sale of 198621 dollars. Corresponding to Twitter and sales data, the fitted regression model is

(3) $$\begin{array}{c} \text{Sales}=5.621+0.193\text{Twitter}. \end{array}$$

The visual display of the relationship between Twitter advertising and the sale of goods is provided in Figure 3. From the plot in Figure 3, it is obvious that there is a positive relationship (PR) between Twitter advertising and sales. The PR means that the more we spend on marketing via the Twitter medium, the more will be the sale.

### 2.2. Statistical Testing

Is there a PR between sales and Twitter advertising medium? Certainly, there is a relationship between them, since the estimated slope *θ*_1_ of the regression line is 5.621, not 0, showing that there is a relationship between sales and Twitter advertisement in the sample of 130 observations. However, we want to know if there is a relationship between the observations of all the sales and Twitter advertisement; that is, we want to know that if *θ*_1_ is unlikely to be 0.

The article "The Role of Twitter Medium in Business with Regression Analysis and Statistical Modelling" was published in 2021. Journal: Comput Intell Neurosci.

For these purposes, we adopt a standard hypothesis approach to conduct a hypothesis test for *θ*_1_. To carry out the procedure, first, we need to accomplish and specify *H*_0_ and *H*_*A*_ as follows: *H*_0_ : *θ*_1_=0 (no significant relationship exists between sales and Twitter advertisement) versus *H*_*A*_ : *θ*_1_ ≠ 0 (a significant relationship exists between sales and Twitter advertisement). Second, we obtain the value of *t*-*statistics* using the following formula:

(4) $$\begin{array}{c} t=\frac{\hat{\theta_{1}}-\theta_{1}}{S.E\left(\hat{\theta_{1}}\right)},\\ t=\frac{\hat{\theta_{1}}-\theta_{1}}{\sqrt{MSE}/\sqrt{\sum_{i=0}^{n}{\left(x_{i}-\bar{x}\right)}^{2}}}. \end{array}$$

Third, we compute the value of *t*-*statistics* using statistical software. By default, the *t*-*statistics* is calculated by assuming that *θ*_1_=0. Divide the estimated coefficient $\hat{\theta_{1}}=5.621$ by its standard error $S.E\hat{\theta_{1}}=0.44428$ to get the value of *t*-*statistics* as follows:

(5) $$\begin{array}{c} t=\frac{5.621-0}{0.44428},\\ t=\frac{5.621}{0.44428},\\ t=12.652. \end{array}$$

Fourth, we calculate the *p* value. By default, the *p* value is calculated by assuming *H*_*A*_ is a “not-equal-to.” If the *p* value is less than 0.05, then we reject *H*_*A*_. After performing the analysis, we observe that the *p* value is 2*e* − 16.

Since the *p* value is very small (less than 0.001), we reject the hypothesis of *θ*_1_=0 and accept the hypothesis of *θ*_1_ ≠ 0. Henceforth, there is significant evidence that there is a linear relationship between sales and Twitter advertisement.

### 2.3. Residuals

The regression line is used to quantify a linear trend in the data. The residual represents the distance between the true value and observed values of *Y*. Mathematically, it is given by

(6) $$\begin{array}{c} \varepsilon =y-\hat{y}. \end{array}$$

The residual standard error is used to quantify the quality of the regression fit. In this study, it represents the average amount of the sales variable (*Y*) varies from the true regression line. In the context of this study, a visual display of the behavior of the residuals is provided in Figure 4.

From the plots presented in Figure 4, we have the following observations:

1. From the residual versus fitted plot, we can see that the red line is quite close to the residual value of 0. Therefore, we assume that the residuals possess the linear property. By linearity, we mean that the *X* in the regression model has a straight-line relationship with *Y*.
2. One of the fundamental assumptions of regression modeling is the normality of the data. The QQ (quantile-quantile) plot makes an angle of 45 showing that the residuals are approximately normally distributed.
3. Homoscedasticity is one of the basic assumptions of linear regression modeling. If this assumption of homoscedasticity does not hold, then the problem of heteroscedasticity arises. The scale-location plot shows that the residuals satisfy the homoscedasticity property.
4. In regression modeling, the influential observations have a serious effect on the parameters estimates. The residual versus leverage plot shows that there are fewer influential observations in the data.

The article "The Role of Twitter Medium in Business with Regression Analysis and Statistical Modelling" was published in 2021. Journal: Comput Intell Neurosci.

### 2.4. Correlation Test

A correlation test is a statistical tool used to quantify the relationship between two or more variables. In this study, we have only two variables (sales and Twitter advertising). Henceforth, we adopt the Pearson correlation approach, which is used to measures a linear relationship between two variables. The coefficient of the Pearson correlation is usually denoted by *r* and derived as

(7) $$\begin{array}{c} r=\frac{\sum_{k=1}^{130}\left(\text{Twitter}-\mu_{\text{Twitter}}\right)\left(\text{Sales}-\mu_{\text{Sales}}\right)}{\sqrt{\sum_{k=1}^{130}{\left(\text{Twitter}-\mu_{\text{Twitter}}\right)}^{2}{\left(\text{Sales}-\mu_{\text{Sales}}\right)}^{2}}}, \end{array}$$

where *μ*_Twitter_ and *μ*_Sales_ represent the mean values of Twitter and sales, respectively. The significance of *r* can be tested by using the *t*-test and is given by

(8) $$\begin{array}{c} t=\frac{r}{\sqrt{1-r^{2}}}\sqrt{n-2}. \end{array}$$

To the test *r*, we use the hypothesis procedure as *H*_0_=0 (there is no relationship between Twitter advertising and sale) versus *H*_*A*_ ≠ 0. After performing the required steps of analysis, we observe that *r*=0.5253, showing a positive relationship between sales and Twitter advertising. Furthermore, we observe that the Spearman rank correlation test represented by *Sp*, is 161 with *p* value given by 4.634*e* − 12. As we see that *p*-value < 0.05, we reject *H*_0_ and conclude that there is a significant relationship between Twitter advertising and sale. This relationship has also been shown graphically in Figure 5.

### 2.5. Testing of Normality

As we stated above that in the domain of regression modeling, the assessment of the normality of data is one of the basic requirements. Basically, there are two approaches for testing the normality of the data: (i) numerically and (ii) graphically. For numerical analysis, we use the Shapiro–Wilk (SW) test for checking the normality of the sales and Twitter advertising data. This test is carried out in the following manner, *H*_0_= the sale data is not normally distributed versus *H*_*A*_= the sale data is normally distributed. After applying the SW test, we found that (i) for the Twitter advertising data, SW=0.96011 with *p* value =0.000739 and (ii) for the sale data, SW=0.967900 with *p* value =0.00356.

The article "The Role of Twitter Medium in Business with Regression Analysis and Statistical Modelling" was published in 2021. Journal: Comput Intell Neurosci.

Since the *p* values associated with the Twitter advertising data and sales data are less than 0.05, we reject *H*_0_ and accept the assumption of normality.

In addition to the numerical test (SW test), we also use a visual approach based on the QQ plot; see Figure 6. For assuming the normality, the QQ plot makes an angle of 45 degrees. Since all the data points are scattered around the referenced line, we can say that the sales and Twitter advertising data sets are normally distributed.

## 3. Statistical Modeling

This section consists of four sections: (i) in the very first section, we describe how the new model is obtained, (ii) in the second section, the proposed model is introduced and its different PDF (probability density function) plots are sketched, (iii) in the third section, we discuss the regularly varying tail behavior of the proposed model, and (iv) finally, a real application is discussed in the last section.

### 3.1. Development of the New Model

Before investing in a particular domain, it is always of interest to have the best description of that domain. The statistical distributions play a great role in describing the phenomena under consideration. Among the statistical distributions in the available literature, the EE (exponentiated exponential) model applied as an alternative to the two-parameter Weibull and Gamma distributions, has attracted many researchers. The DF (distribution function) of the EE model expressed by *H*(*y*; Φ) is

(9) $$\begin{array}{c} H\left(y;\Phi \right)={\left(1-\exp\left\{-\delta_{2}y\right\}\right)}^{\delta_{1}},\;y\geq 0,\delta_{1},\delta_{2}>0, \end{array}$$

where *δ*_1_ is a shape and *δ*_2_ is the scale parameter of the EE distribution. The PDF (probability density function) of the EE model represented by *h*(*y*; Φ) is

(10) $$\begin{array}{c} h\left(y;\Phi \right)=\delta_{1}\delta_{2}\exp\left\{-\delta_{2}y\right\}{\left(1-\exp\left\{-\delta_{2}y\right\}\right)}^{\delta_{1}-1},\;y>0. \end{array}$$

As we know in the finance sector, the data sets, particularly the financial returns, are frequently right-skewed with heavy tails. Among the class of statistical distributions, the HT distributions have shown better performance in modeling data in the finance sector where the financial returns experience HT, right-skewed, and unimodal behavior. According to Beirlant et al. [11], a model is called HT distribution, its SF (survival function) $\bar{H}\left(y;\Phi \right)=1-H\left(y;\Phi \right)$, satisfies

(11) $$\begin{array}{c} \underset{y⟶\infty }{\lim}=\exp\left\{ay\right\}H\left(y;\Phi \right)=\infty , \end{array}$$

where *a* > 0.

The article "The Role of Twitter Medium in Business with Regression Analysis and Statistical Modelling" was published in 2021. Journal: Comput Intell Neurosci.

An important characteristic of the HT distributions is the RVP (regular variational property); see Resnick [12]. A model is called RVD (regular varying distribution) if it satisfies

(12) $$\begin{array}{c} \underset{y⟶\infty }{\lim}\frac{1-H\left(uy;\Phi \right)}{1-H\left(y;\Phi \right)}=u^{-a},\;a\in \left\{0,\infty \right\}. \end{array}$$

The distributions which possess the RVP are very useful models for dealing with the financial returns and HT data; see [13], [14], [15], and [16].Numerous methods to obtain new HT and flexible distributions have been introduced. Among the available methods in the literature, the exponential TX family is a prominent method to generate HT distributions [17]. For *σ* > 1 and *y* ∈ *ℝ*, the DF *G*(*y*; Φ), and PDF *g*(*y*; Φ) of the exponential TX family are given by

(13) $$\begin{array}{c} G\left(y;\Phi \right)=1-\frac{\sigma \bar{H}\left(y;\Phi \right)}{\sigma -H\left(y;\Phi \right)}, \end{array}$$

(14) $$\begin{array}{c} g\left(y;\Phi \right)=\frac{\sigma \left(\sigma -1\right)h\left(y;\Phi \right)}{{\left(\sigma -H\left(y;\Phi \right)\right)}^{2}}. \end{array}$$

Keeping in view the role of the HT distributions in the finance sectors, we are motivated to study a new HT model called ETXE-exponential distribution. The ETXE-exponential distribution is obtained by incorporating equation (1) in equation (13).

The ETXE-exponential distribution is very interesting and offers to model the data that are skewed to right with a heavy tail. This fact is shown in the coming three sections. For example, the graphical behavior of its PDF is shown in section 3.2, where we can see that the ETXE-exponential distribution is a HT model. Secondly, the HT properties of the ETXE-exponential distribution are proved in section 3.3. Finally, positively skewed data related to the sales are analyzed in section 3.4, where we show that the ETXE-exponential distribution can be a better model for the HT financial data sets as compared to other existing distributions.

### 3.2. The ETXE-Exponential Distribution

A random variable *Y* has the ETXE-exponential model with scale parameters *δ*_2_ > 0, *σ* > 1 and shape parameter *δ*_1_ > 0, if its DF is

(15) $$\begin{array}{c} G\left(y;\Phi \right)=1-\frac{\sigma \left(1-{\left(1-\exp\left\{-\delta_{2}y\right\}\right)}^{\delta_{1}}\right)}{\sigma -{\left(1-\exp\left\{-\delta_{2}y\right\}\right)}^{\delta_{1}}},\;y\geq 0, \end{array}$$

and PDF is

(16) $$\begin{array}{c} g\left(y;\Phi \right)=\frac{\delta_{1}\delta_{2}\sigma \left(\sigma -1\right)\exp\left\{-\delta_{2}y\right\}{\left(1-\exp\left\{-\delta_{2}y\right\}\right)}^{\delta_{1}-1}}{{\left(\sigma -{\left(1-\exp\left\{-\delta_{2}y\right\}\right)}^{\delta_{1}}\right)}^{2}},\;y>0. \end{array}$$

Some possible behaviors of *g*(*y*; Φ) are sketched in Figure 7. The plots of *g*(*y*; Φ) in Figure 7 (left panel), are sketched for *δ*_1_=1.2, *δ*_2_=0.8, *σ*=1.8 (red line); *δ*_1_=2.8, *δ*_2_=0.8, *σ*=1.8 (green line); and *δ*_1_=4.8, *δ*_2_=0.8, *σ*=1.8 (black line), whereas the plots of *g*(*y*; Φ) in Figure 7 (right panel) are sketched for *δ*_1_=1.2, *δ*_2_=0.8, *σ*=1.2 (red line); *δ*_1_=1.2, *δ*_2_=0.8, *σ*=1.8 (green line); and *δ*_1_=1.2, *δ*_2_=0.8, *σ*=2.5 (black line).

The article "The Role of Twitter Medium in Business with Regression Analysis and Statistical Modelling" was published in 2021. Journal: Comput Intell Neurosci.

From the PDF plots sketched in Figure 7 (left panel), it is clear that when the value of *δ*_1_ increases, the ETXE-exponential distribution tends to a HT distribution. Also, from the PDF plots sketched in Figure 7 (right panel), as the value of *σ* increases the proposed EXTE-exponential distribution possesses HT behavior.

### 3.3. The Heavy-Tailed Behavior

This section deals with the regularly varying tail behavior of the ETXE-exponential distribution which is very important to characterize the HT property of a model.

#### 3.3.1. The Regularly Varying Tail Behavior

According to Karamata's theorem [18], in terms of SF (survival function) $\bar{G}\left(y;\Phi \right)$, we have the following.

**Theorem 1 .**

If $\bar{H}\left(y;\Phi \right)\left(\right)$ is the SF of the RVD, then $\bar{G}\left(y;\sigma ,\Phi \right)$ is a RVD.

**Proof**

Suppose$\lim_{y⟶\infty }\bar{H}\left(ky;\Phi \right)/\bar{H}\left(y;\Phi \right)=g\left(k\right)$ is finite but nonzero for every *k* > 0. Using equation (3), we have

(17) $$\begin{array}{c} \underset{y⟶\infty }{\lim}\;\frac{\bar{G}\left(ky;\sigma ,\Phi \right)}{\bar{G}y;\sigma ,\Phi }=\underset{y⟶\infty }{\lim}\;\frac{\sigma \bar{H}\left(ky;\Phi \right)}{\sigma \bar{H}\left(y;\Phi \right)}\cdot \frac{\sigma -H\left(y;\Phi \right)}{\sigma -H\left(ky;\Phi \right)}. \end{array}$$

Using equation (1) in equation (17), we get

(18) $$\begin{array}{c} \underset{y⟶\infty }{\lim}\;\frac{\bar{G}\left(ky;\sigma ,\Phi \right)}{\bar{G}\left(y;\sigma ,\Phi \right)}=\underset{y⟶\infty }{\lim}\frac{\sigma \bar{H}\left(ky;\Phi \right)}{\sigma \bar{H}\left(y;\Phi \right)}\cdot \frac{\sigma -{\left(1-\exp\left\{-\delta_{2}y\right\}\right)}^{\delta_{1}}}{\sigma -{\left(1-\exp\left\{-\delta_{2}y\right\}\right)}^{\delta_{1}}},\\ \underset{y⟶\infty }{\lim}\frac{\bar{G}\left(ky;\sigma ,\Phi \right)}{\bar{G}\left(y;\sigma ,\Phi \right)}=\underset{y⟶\infty }{\lim}\frac{\sigma \bar{H}\left(ky;\Phi \right)}{\sigma \bar{H}\left(y;\Phi \right)}\cdot \frac{\sigma -{\left(1-\exp\left\{-\delta_{2}\infty \right\}\right)}^{\delta_{1}}}{\sigma -{\left(1-\exp\left\{-\delta_{2}\infty \right\}\right)}^{\delta_{1}}},\\ \underset{y⟶\infty }{\lim}\frac{\bar{G}\left(ky;\sigma ,\Phi \right)}{\bar{G}\left(y;\sigma ,\Phi \right)}=\underset{y⟶\infty }{\lim}\frac{\sigma \bar{H}\left(ky;\Phi \right)}{\sigma \bar{H}\left(y;\Phi \right)}\cdot \frac{\sigma -{\left(1-\exp\left\{\infty \right\}\right)}^{\delta_{1}}}{\sigma -{\left(1-\exp\left\{-\infty \right\}\right)}^{\delta_{1}}},\\ \underset{y⟶\infty }{\lim}\frac{\bar{G}\left(ky;\sigma ,\Phi \right)}{\bar{G}\left(y;\sigma ,\Phi \right)}=\underset{y⟶\infty }{\lim}\frac{\sigma \bar{H}\left(ky;\Phi \right)}{\sigma \bar{H}\left(y;\Phi \right)}\cdot \frac{\sigma -{\left(1-0\right)}^{\delta_{1}}}{\sigma -{\left(1-0\right)}^{\delta_{1}}},\\ \underset{y⟶\infty }{\lim}\frac{\bar{G}\left(ky;\sigma ,\Phi \right)}{\bar{G}\left(y;\sigma ,\Phi \right)}=\underset{y⟶\infty }{\lim}\frac{\sigma \bar{H}\left(ky;\Phi \right)}{\sigma \bar{H}\left(y;\Phi \right)}\cdot \frac{\sigma -1}{\sigma -1},\\ \underset{y⟶\infty }{\lim}\frac{\bar{G}\left(ky;\sigma ,\Phi \right)}{\bar{G}\left(y;\sigma ,\Phi \right)}=\underset{y⟶\infty }{\lim}\frac{\sigma \bar{H}\left(ky;\Phi \right)}{\sigma \bar{H}\left(y;\Phi \right)},\\ \underset{y⟶\infty }{\lim}\frac{\bar{G}\left(ky;\sigma ,\Phi \right)}{\bar{G}\left(y;\sigma ,\Phi \right)}=g\left(k\right), \end{array}$$

which is finite but nonzero for every *k* > 0; thus, $\bar{G}\left(y;\sigma ,\Phi \right)$ is a RVD.

The article "The Role of Twitter Medium in Business with Regression Analysis and Statistical Modelling" was published in 2021. Journal: Comput Intell Neurosci.

#### 3.3.2. An Application of the Regularly Varying Tail Behavior

Let us assume that the distribution of *Y* has PLB (power law behavior); then, we have

(19) $$\begin{array}{c} 1-H\left(y;\Phi \right)=\bar{H}\left(y;\Phi \right)=\mathbb{P}\left(Y>y\right)∼y^{-\beta }. \end{array}$$

Utilizing Karamata's theorem [18], we can write $\bar{G}\left(y;\Phi \right)$ as

(20) $$\begin{array}{c} \bar{G}\left(y;\Phi \right)=y^{-\beta }L\left(y;\Phi \right), \end{array}$$

where *L*(*y*; Φ) is slowly varying. Note that

(21) $$\begin{array}{c} \bar{G}\left(y;\Phi \right)=\frac{\sigma \bar{H}\left(y;\Phi \right)}{\sigma -1+\bar{H}\left(y;\Phi \right)}. \end{array}$$

Since $\bar{H}\left(y;\Phi \right)∼y^{-\beta }$, we can write

(22) $$\begin{array}{c} \bar{G}\left(y;\Phi \right)=\frac{\sigma y^{-\beta }}{\sigma -1+y^{-\beta }}=y^{-\beta }L\left(y;\Phi \right), \end{array}$$

where *L*(*y*; Φ)=*σ*/*σ* − 1+*y*^−*β*^. If *L*(*y*; Φ) is a SVF (slowly varying function), then the variational result obtained is true. As per Resnick [12], for all *β* > 0, we have to show that

(23) $$\begin{array}{c} \underset{y⟶\infty }{\lim}\frac{L\left(\beta y;\Phi \right)}{L\left(y;\Phi \right)}=1. \end{array}$$

After some computation, we get

(24) $$\begin{array}{c} \frac{L\left(by;\Phi \right)}{L\left(y;\Phi \right)}=\frac{\sigma \left(\sigma -1+\left(1/y^{\beta }\right)\right)}{\sigma \left(\sigma -1+\left(1/y^{\beta }b^{\beta }\right)\right)}. \end{array}$$

If *y*⟶*∞*, then lim_*y*⟶*∞*_(1/*y*^*β*^)=0, and lim_*y*⟶*∞*_(1/*y*^*β*^*b*^*β*^)=0. Therefore, from equation (14), we have

(25) $$\begin{array}{c} \frac{L\left(by;\Phi \right)}{L\left(y;\Phi \right)}=\frac{\sigma \left(\sigma -1\right)}{\sigma \left(\sigma -1\right)}. \end{array}$$

Finally, we get the required result

(26) $$\begin{array}{c} \underset{y⟶\infty }{\lim}\frac{L\left(by;\Phi \right)}{L\left(y;\Phi \right)}=1. \end{array}$$

### 3.4. Analyzing the Sales Data

As we mentioned earlier that the HT statistical models are very useful in describing the financial phenomena. In this section, we show the best fitting power of the ETXE-exponential model via analyzing the sales data which is consists of 130 observations. The Twitter advertising and sales data sets are available at https://data.world/datasets/twitter.  Table 1 offers the BMs (basic measures) of the sales data.

The total time test (TTT), histogram, and box plot of the sales data are provided in Figure 8. From Figure 8, we can easily observe that the data set is unimodal and skewed to the right. The data set possessing such characteristics can be better modeled via using the ETXE-exponential distribution.

The comparison of the ETXE-exponential is made with three well-known distributions available in the literature. The DFs of the competing models are as follows:

(1) MOW (Marshall–Olkin Weibull) model [19]:
  (27) $$\begin{array}{c} H\left(y;\Phi \right)=1-\frac{\sigma e^{-\delta_{2}y^{\delta_{1}}}}{\left(1-\left(1-\sigma \right)e^{-\delta_{2}y^{\delta_{1}}}\right)},\;y\geq 0,\sigma ,\delta_{1},\delta_{2}>0. \end{array}$$
(2) FW (flexible Weibull) model [20]:
  (28) $$\begin{array}{c} H\left(y;\Phi \right)=1-e^{-e^{\left(\gamma y\left(\beta /y\right)-\right)}},\;y\geq 0,\gamma ,\beta >0. \end{array}$$
(3) APTW (alpha power transformed Weibull) model [21]:
  (29) $$\begin{array}{c} H\left(y;\Phi \right)=\frac{\alpha^{1-e^{-\delta_{2}y^{\delta_{1}}}}-1}{\alpha -1},\;y\geq 0,\alpha ,\delta_{1},\delta_{2}>0,\alpha \neq 1. \end{array}$$
The term “better modeling” is used in the sense that the ETXE-exponential distribution has the smaller values of the selected IC (information criterion) considered for comparison. The expressions of the IC are given by the following:
(4) The AIC (Akaike IC) [22] is
  (30) $$\begin{array}{c} \text{AIC}=2k-2\ell . \end{array}$$
(5) The BIC (Bayesian IC) [23] is
  (31) $$\begin{array}{c} \text{BIC}=k\;\log\left(n\right)-2\ell . \end{array}$$
(6) The HQIC (Hannan-Quinn IC) [24] is
  (32) $$\begin{array}{c} \text{HQIC}=2k\;\log\left(\log\left(n\right)\right)-2\ell . \end{array}$$
(7) The CAIC (Corrected Akaike IC) [25] is
  (33) $$\begin{array}{c} \text{CAIC}=\frac{2nk}{n-k-1}-2\ell . \end{array}$$

In addition to the IC, we further considered three goodness of fit measures (g-o-f) including the following:

(1) The AD (Anderson–Darling) test statistic:
  (34) $$\begin{array}{c} \text{AD}=-k-\frac{1}{k}\sum_{u=1}^{k}\left(2u-1\right)\left[\log\;H\left(y_{u}\right)+\log\left\{1-H\left(y_{k-u+1}\right)\right\}\right]. \end{array}$$
(2) The CM (Cramer–von Mises) test statistic:
  (35) $$\begin{array}{c} \text{CM}=\frac{1}{12k}+\sum_{u=1}^{k}{\left[\frac{2u-1}{2k}-H\left(y_{u}\right)\right]}^{2}. \end{array}$$
(3) The KS (Kolmogorov–Smirnov (KS) test statistic:

(36) $$\begin{array}{c} \text{KS}=\underset{y}{\text{sup}}\left[H_{k}\left(y\right)-H\left(y\right)\right]. \end{array}$$

The optimization technique is adopted to get the MLEs (maximum likelihood estimators) of the competing models. In this section, we implement the Newton–Raphson (NR) iteration approach to get the MLEs of the fitted models using the sales data. The MLEs of the fitted models are provided in Table 2. The values of the IC are reported in Table 3, and the g-o-f measures with *p* value are presented in Table 4.

The article "The Role of Twitter Medium in Business with Regression Analysis and Statistical Modelling" was published in 2021. Journal: Comput Intell Neurosci.

Based on the sales data, the results reported in Tables 3 and 4, we can see that the ETXE-exponential distribution has the smallest values of the IC and g-o-f measures. The values of the selected measures for the ETXE-exponential distribution are IC = 0.0237, CAIC = 0.2027, BIC = 0.0336, HQIC = 0.9985, AD = 0.0237, CM = 0.2027, KS 0.0336, and *p* value = 0.9985. For the second-best competitive model (FW distribution), these measures are AIC = 648.4654, CAIC = 648.5599, BIC = 654.2005, HQIC = 650.7957, AD = 0.0719, CM = 0.4315, KS = 0.0861, and *p* value = 0.2896. We can see that the FW is the second-best model, but not in terms of KS and *p* value. From Table 4, it is clear that the APTW distribution is the second-best model as it has the second smallest KS value which is 0.0559, and the second-highest *p* value which is 0.8106.

Furthermore, for the best description of the results of the sales data, the estimated PDF and CDF plots of the fitted models (EXTE-exponential (red line), MOW (green line), APTW (pink line), and FW (blue line)) are provided in Figure 9. The PP (probability-probability), and QQ plots are sketched in Figures 10 and 11, respectively.

## 4. Future Research Directions

In this work, we restricted our study to simple linear regression analysis by using the Twitter medium as a predictor variable. However, many other online mediums can be used for advertising purposes such as YouTube, Facebook, and Twitter. Therefore, in the future, we are intended to implement the multiple linear regression modeling approach to see the impact of different advertising mediums on sales. Generally, the multiple linear regression model (MLRM) with *k* predictors is given by

(37) $$\begin{array}{c} Y=\theta_{0}+\theta_{1}X_{1}+\theta_{2}X_{2}+\theta_{3}X_{3}+,\ldots ,\theta_{k}X_{k}+\varepsilon . \end{array}$$

The future research study will be carried out in three different phases. For example, (i) in phase one, the MLRM will be implemented with two (*X*_1_= medium 1, *X*_2_  = medium 2) advertising mediums; (ii) in phase two, the MLRM will be used by considering three (*X*_1_=medium 1, *X*_2_  = medium 2, *X*_3_  = medium 3) advertising mediums; and (iii) in phase three, the MLRM will be applied by taking four (*X*_1_=medium 1, *X*_2_  = medium 2, *X*_3_  = medium 3, *X*_4_  = medium 4) advertising mediums.

### 4.1. The MLRM with Two Predictors

The MLRM with two predictors is given by

(38) $$\begin{array}{c} Y=\theta_{0}+\theta_{1}X_{1}+\theta_{2}X_{2}+\varepsilon . \end{array}$$

In the future, we are planning to use the MLRM defined in equation (38) to see the impact of two different advertising mediums on sales. The MLRM models with possible combinations of two different advertising mediums are given by the following:

(1) Effect of Twitter and YouTube advertising mediums on sales
The MLRM with two advertising mediums (*X*_1_=Twitter and *X*_2_ = YouTube) is given by
  (39) $$\begin{array}{c} \text{Sales}=\theta_{0}+\theta_{1}\text{Twitter}+\theta_{2}\text{YouTube}+\varepsilon . \end{array}$$
(2) Effect of Twitter and Facebook advertising mediums on sales
The MLRM with two advertising mediums (*X*_1_=Twitter and *X*_2_ = Facebook) is given by
  (40) $$\begin{array}{c} \text{Sales}=\theta_{0}+\theta_{1}\text{Twitter}+\theta_{2}\text{Facebook}+\varepsilon . \end{array}$$
(3) Effect of Twitter and Instagram advertising mediums on sales.
The MLRM with two advertising mediums (*X*_1_=Twitter and *X*_2_ = Instagram) is given by
  (41) $$\begin{array}{c} \text{Sales}=\theta_{0}+\theta_{1}\text{Twitter}+\theta_{2}\text{Instagram}+\varepsilon . \end{array}$$

The article "The Role of Twitter Medium in Business with Regression Analysis and Statistical Modelling" was published in 2021. Journal: Comput Intell Neurosci.

### 4.2. The MLRM with Three Predictors

The MLRM with three predictors is given by

(42) $$\begin{array}{c} Y=\theta_{0}+\theta_{1}X_{1}+\theta_{2}X_{2}+\theta_{3}X_{3}+\varepsilon . \end{array}$$

In the future, we are also interested in using the MLRM defined in equation (42) to see the impact of three different advertising mediums on sales. The MLRM models with possible combinations of three different advertising mediums are given by the following:

(1) Effect of Twitter, YouTube, and Facebook advertising mediums on sales.
The MLRM with three different advertising mediums (*X*_1_=Twitter, *X*_2_ = YouTube, *X*_3_ = Facebook) is given by
  (43) $$\begin{array}{c} \text{Sales}=\theta_{0}+\theta_{1}\text{Twitter}+\theta_{2}\text{YouTube}+\theta_{3}\text{Facebook}+\varepsilon . \end{array}$$
(2) Effect of Twitter, YouTube, and Instagram advertising mediums on sales.
The MLRM with three different advertising mediums (*X*_1_=Twitter, *X*_2_ = YouTube, *X*_3_ = Instagram) is given by
  (44) $$\begin{array}{c} \text{Sales}=\theta_{0}+\theta_{1}\text{Twitter}+\theta_{2}\text{YouTube}+\theta_{3}\text{Instagram}+\varepsilon . \end{array}$$

### 4.3. The MLRM with Four Predictors

The MLRM with four predictors is given by

(45) $$\begin{array}{c} Y=\theta_{0}+\theta_{1}X_{1}+\theta_{2}X_{2}+\theta_{3}X_{3}+\theta_{4}X_{4}+\varepsilon . \end{array}$$

In the future, we are also motivated to use the MLRM defined in equation (45) to see the impact of four different advertising mediums on sales.

(1) Effect of Twitter, YouTube, Facebook, and Instagram advertising mediums on sales
The MLRM with four different advertising mediums (*X*_1_=Twitter, *X*_2_ = YouTube, *X*_3_ = Facebook, *X*_4_ = Instagram) is given by
  (46) $$\begin{array}{c} \text{Sales}=\theta_{0}+\theta_{1}\text{Twitter}+\theta_{2}\text{YouTube}+\theta_{3}\text{Facebook}+\theta_{3}\text{Instagram}+\varepsilon . \end{array}$$

## 5. Concluding Remarks

In this research, we studied the relationship between Twitter advertising and sales by adopting the simple linear regression approach. For testing the impact of Twitter medium as an advertising tool, two main statistical approaches such as *t*-test and correlation test are utilized. Based on the results of the *t*-test and correlation test, it is observed that Twitter advertising plays a useful role in increasing sales. Furthermore, a new HT model called the ETXE-exponential distribution is developed by combining the exponentiated-exponential model with the ETX family. The ETXE-exponential distribution was introduced to provide a close fit to sales data, which is an important area of the finance sector. For proving the applicability of the proposed model, the sales data is analyzed. The comparison of the ETXE-exponential distribution was made with MOW, APTW, and FW distributions. By taking into account certain analytical tools, we showed that the ETXE-exponential distribution is the best model for modeling data in the finance sector.

The article "The Role of Twitter Medium in Business with Regression Analysis and Statistical Modelling" was published in 2021. Journal: Comput Intell Neurosci.

## Figures and Tables

**Figure 1:** Leading social media platforms used by the business community around the globe in 2020.

**Figure 2:** Main division of the regression modeling.

**Figure 3:** Graphical display of the relationship between Twitter advertising and sales.

**Figure 4:** Graphical sketching of the residuals behaviors.

**Figure 5:** Visual display of the correlation test results.

**Figure 6:** Graphical display of the SW tests result for the Twitter advertising and sale data.

**Figure 7:** Different PDF plots of the ETXE-exponential distribution.

**Figure 8:** The TTT, histogram, and box plots for the sales data.

**Figure 9:** The estimated PDF, CDF, and KMS plots of the fitted distributions.

**Figure 10:** The PP plots of the fitted distributions.

**Figure 11:** The QQ plots of the fitted distributions.

**Table 1:** The SMs of the sales data.

Observations	Min.	1^st^ Qu.	Median	Mean	3_rd_ Qu.	Max.
130	2.691	6.167	7.997	8.310	10.091	19.777

**Table 2:** The MLEs of the fitted models.

Models	*δ*_1_	*δ*_2_	*σ*	*α*	*γ*	*β*
ETXE-exponential	13.6215	0.4655	1.7019	—	—	—
MOW	2.6988	0.0030	1.4851	—	—	—
APTW	1.8410	0.0367	—	44.6860	—	—
FW	—	—	—	—	0.1482	13.0846

**Table 3:** The IC of the fitted models.

Models	AIC	CAIC	BIC	HQIC
ETXE-exponential	644.9836	645.1741	653.5862	648.4791
MOW	655.2653	655.4558	663.8679	658.7608
APTW	651.5548	651.7453	660.1574	655.0503
FW	648.4654	648.5599	654.2005	650.7957

**Table 4:** The goodness of fit measures of the fitted models.

Models	AD	CM	KS	*p* value
ETXE-exponential	0.0237	0.2027	0.0336	0.9985
MOW	0.1433	0.8511	0.0773	0.4188
APTW	0.0912	0.5847	0.0559	0.8106
FW	0.0719	0.4315	0.0861	0.2896

## Data Availability

The data are available from the corresponding author upon request.
